# Evaluation of Resilient Modulus of Subgrade and Base Materials in Indiana and Its Implementation in MEPDG

**DOI:** 10.1155/2014/372838

**Published:** 2014-02-20

**Authors:** Richard Ji, Nayyarzia Siddiki, Tommy Nantung, Daehyeon Kim

**Affiliations:** ^1^INDOT Office of Research and Development, 1205 Montgomery Street, West Lafayette, IN 47906, USA; ^2^INDOT Materials and Testing, 100 N. Senate Avenue, Indianapolis, IN 46204, USA; ^3^Department of Civil Engineering, Chosun University, 375 Seosuk-Dong, Dong-Gu, Gwangju 501-759, Republic of Korea

## Abstract

In order to implement MEPDG hierarchical inputs for unbound and subgrade soil, a database containing subgrade *M*_*R*_, index properties, standard proctor, and laboratory *M*_*R*_ for 140 undisturbed roadbed soil samples from six different districts in Indiana was created. The *M*_*R*_ data were categorized in accordance with the AASHTO soil classifications and divided into several groups. Based on each group, this study develops statistical analysis and evaluation datasets to validate these models. Stress-based regression models were evaluated using a statistical tool (analysis of variance (ANOVA)) and *Z*-test, and pertinent material constants (*k*_1_, *k*_2_ and *k*_3_) were determined for different soil types. The reasonably good correlations of material constants along with *M*_*R*_ with routine soil properties were established. Furthermore, FWD tests were conducted on several Indiana highways in different seasons, and laboratory resilient modulus tests were performed on the subgrade soils that were collected from the falling weight deflectometer (FWD) test sites. A comparison was made of the resilient moduli obtained from the laboratory resilient modulus tests with those from the FWD tests. Correlations between the laboratory resilient modulus and the FWD modulus were developed and are discussed in this paper.

## 1. Background

Resilient modulus (*M*_*R*_) is an important mechanical property widely used for the analysis and design of pavements. Therefore the determination of the resilient modulus of pavement materials is of vital importance for any mechanistically based design/analysis procedure for pavements. In the past, the Indiana Department of Transportation's (INDOT's) flexible and rigid pavement design process followed the procedures outlined in the 1993 American Association of State Highway and Transportation Officials (AASHTO) *Guide for Design of Pavement Structures* (Design Guide) [1]. One of the inputs of these procedures is the effective value of the resilient modulus of the roadbed soil, which is a function of seasonal changes, soil type, moisture content, and testing method.

The *Mechanistic-Empirical Design Guide* (MEPDG) [2] requires the resilient modulus of unbound and cohesive soil materials to characterize layers for their structural design. Moisture and temperature variations within the pavement structure are calculated internally using the Enhanced Integrated Climatic Model (EICM). Level 1 requires material constants (*k*_1_, *k*_2_, and *k*_3_) from actual *M*_*R*_ testing data. The level 2 design uses correlations to determine *M*_*R*_ soil properties and gives intermediate reliability. *M*_*R*_ values are estimated from correlations with the soil index and other properties such as CBR or layer coefficient. The required design data inputs for level 2 could be selected from an agency database, derived from a limited testing program, or estimated through correlations. Level 3, the lowest reliability level, uses default values based on soil classifications. Several departments of transportation (DOTs) have already created or are in the process of creating *M*_*R*_ databases for local soils. These agencies have found their *M*_*R*_ databases to be very useful tools for improving pavement designs and analyses using the MEPDG [3, 4].

It is known that a laboratory resilient modus test and a falling weight deflectometer (FWD) test are usually used to obtain the resilient modulus of subgrade [5, 6]. However, the difference between the resilient moduli obtained from these two methods is considerably large due to the fact that these tests are conducted under different conditions. This difference causes engineers significant confusion about how to appropriately input the resilient modulus in the MEPDG software. A successful implementation of the MEPGD requires a comprehensive *M*_*R*_ database for local subgrade soils and its assessment to determine desired input parameters. Thus, it is imperative to evaluate *M*_*R*_ values obtained from the different procedures and ascertain the influence of procedural choice on the design thickness of pavement layers. Since INDOT adopted the MEPDG [2] in January 2009, a database containing subgrade *M*_*R*_, index properties, standard proctor, and cyclic load triaxial test data for 140 soil samples from six different districts in Indiana was developed. On the course of implementation in INDOT, Kim and Siddiki [7] assessed 14 cohesive subgrade soils in Indiana by conducting *M*_*R*_, unconfined compressive strength (UCS), standard proctor, dynamic cone penetration (DCP), and other routine soil tests. They also proposed a regression model based on the UCS tests to estimate the *M*_*R*_, and they developed a predictive model to estimate *k*_1_, *k*_2_, and *k*_3_. Furthermore, Kim et al. [8] evaluated seasonal variations and compared these variations using backcalculated in situ modulus.

## 2. Objectives and Scope

The primary objective of this study was to implement MEPDG with the laboratory test procedure for measuring the resilient modulus of unbound base/subbase materials and subgrade soils in Indiana and to determine whether hierarchical design levels of MEPDG inputs should be fully incorporated into the INDOT design procedure. A secondary objective of this research was to determine the correlations between the modulus from the FWD test and the *M*_*R*_ from the laboratory resilient modulus test by comparing the results obtained from the FWD test on subgrade with those obtained from the laboratory cyclic load triaxial resilient modulus test on subgrade soil samples molded at the optimum moisture content (OMC) in Indiana. A third objective of this research was to provide a catalog of *M*_*R*_ values for base and subgrade materials used in Indiana. Specific objectives included the following.

- Conduct a pilot study for implementing the resilient modulus in the Indiana pavement design procedure.
- Establish procedures (equations) for obtaining the resilient modulus of the roadbed soils for level 1, 2, and 3 designs of the MEPDG.
- Conduct laboratory tests to determine the physical and mechanistic characteristics of the various roadbed soils for Indiana.
- Determine the resilient modulus of the roadbed soils using cyclic load triaxial testing (CTT) in the laboratory and nondestructive deflection test data.
- Evaluate testing methods for determining the resilient modulus on subgrade soils and untreated base/subbase materials for pavement design.
- Correlate laboratory resilient modulus measurements with FWD test results on subgrade soils and untreated base/subbase materials.

## 3. Research Approach

Unbound and subgrade materials are categorized by grain size distribution, liquid limit, and plasticity index value. The designer selects the primary unbound material type using one of the classification systems and then provides further input to determine appropriate material properties to be used for design. The primary input parameter used for design is the resilient modulus. For level 1 design, the resilient modulus values of unbound granular materials, subgrade, and bedrock are determined from triaxial tests (AASHTO T307) [9]. Unbound and subgrade materials can be either stress hardening or stress softening and, therefore, the nonlinear behavior of the material must be established for design. For level 2 designs, the test correlation used to characterize the resilient modulus behavior of unbound materials is described in NCHRP 1-37A [2]; it includes California bearing ratio (CBR), resistance value (*R*-value), DCP, and others.

For level 3 design, the resilient modulus of unbound materials is selected based on the unbound material classification (AASHTO or USC (US Code)). The Design Guide provides a general range of typical modulus values for each unbound material classification at its optimum moisture content. Other important parameters of unbound materials considered by the Design Guide include Atterberg limits, grain size distribution, and moisture/density.

### 3.1. Fine Grain Soil Sampling and Testing

The collected database contains 140 data records representing all classes of soils prescribed by AASHTO. Based on AASHTO classification, the fine grain soil group includes A-4, A-6, and A-7-6 soils. A-1, A-2-4, and A-3 soils are considered to be granular materials and are not commonly encountered in Indiana. Thus, only the representative fine grain soils of the subgrade materials were obtained and transported to the laboratory. INDOT's Materials and Tests Division has historical records of numerous triaxial tests. The basic properties of each soil were evaluated in the laboratory prior to conducting the resilient modulus test. The soils were then reconstituted in the laboratory to match the in situ moisture and density conditions and the optimum conditions for the resilient modulus test. Density was determined by Nuclear Gauge (AASHTO T310) [9] or Sand Cone (AASHTO T191) [9]. Moisture in the field was determined by microwave or stove top (ITM 506). The resilient modulus test method adopted for this project was AASHTO T307-99 [10].

The experimental results from the field plate bearing load and laboratory triaxial resilient modulus tests are presented and discussed in the following sections. For the laboratory triaxial resilient modulus test program, each type of soil was tested under the in situ moisture and density condition and the optimum compacted condition. Before the results from the field and laboratory tests were compared, the difference was examined between the laboratory resilient modulus values under the two moisture and density conditions. The basic properties of test materials for fine grain soils are presented in Table 1, including liquid limit (LL), plastic index (PI), the specific density, the maximum dry unit weight, and the optimum moisture content (OMC).

### 3.2. In Situ Pavement Modeling

In the MEPDG computation models, pavement response computation models incorporated into the mechanistic-empirical design approach require the input of *M*_*R*_ values to represent the stiffness of supporting layers, which include unbound granular base materials and subgrade soils. The MEPDG identifies a three-level hierarchical approach for resilient moduli based on the significance of the project. MEPDG levels 1 and 2 design/analysis require the input of *M*_*R*_ for a given state of stress, which can be determined by performing a layered elastic analysis. AASHTO published AASHTO T307-99 [10], *Determining the Resilient Modulus of Soil and Aggregates Materials*, in which *M*_*R*_ is obtained from the axial deviator stress divided by the recoverable axial strain using a cyclic triaxial load test. The current practice in Indiana to determine *M*_*R*_ from laboratory tests is to specify certain levels of the confining and deviator stresses at a certain number of repeated loading cycles. Since values of *M*_*R*_ vary as a function of stress level, it is important to evaluate the stress levels upon loading. For this purpose, elastic layer analyses for pavement structures with different thickness configurations were performed. The subgrade stress level under the pavement is considered under geostatic and truck loads. The contact area of the modeled truck tire has a nominal radius of 150 mm (5.91 in). It can accurately simulate the in situ unbound soil stress level under FWD testing on asphalt pavement, the 40-kN (9-kip) load of a standard test with a contact pressure of 565.8 kpa (82 psi). The first part is calculated from in situ pressure existing from the pavement system overburden. The second part of the analysis assumes that each layer of pavement is composed of different materials and that the response to loading was calculated based on the resilient modulus (*E*) and Poisson's ratio (*μ*) of the materials. The at-rest earth pressure coefficient is used for this study, because the deformation in the subgrade from imposed wheel loading is usually small. The *k*_0_ for cohesive and noncohesive soils is normally considered to be a function of Poisson's ratio and a function of the angle of internal friction *ϕ*, respectively.

The program KENLAYER was used to calculate stresses in pavements under static loads. The vertical and horizontal stresses were obtained with 40 kN (9 kips) ESAL (equivalent single axle loads), imitating actual traffic conditions:

(1) $$\begin{array}{c} k_{0}=\frac{\nu }{1-\nu }, \end{array}$$

(2) $$\begin{array}{c} k_{0}=1-\sin\phi . \end{array}$$

Since this study involved both granular and cohesive materials, it is assumed that granular materials will be used as the base layer and cohesive material as the subgrade. The stress point considered for the granular base material was located midlayer and the stress point for the subgrade material was located at the top of the subgrade.

A limited sensitivity analysis was also conducted to address the influence of the material strength on stresses under the pavement surface. This study considered a typical asphalt pavement in Indiana. The asphalt layer is usually 101.6 to 203.2 mm (4 to 8 in) thick over a 203.2 to 304.8 mm (8 to 12 in) aggregate base. The configuration of the pavement used and the modulus for the base layer and subgrade are shown in Table 2. Figures 1 and 2 summarize the stress level results due to truck and overburden loading. This configuration yields a deviator pressure of approximately 27.6 to 55.2 kPa (4 to 8 psi) confining stress and a deviator stress of 89.7 to 110.4 kPa (13 to 16 psi) for the base. The stress level in subgrade yields a deviator stress of 41.4 to 48.3 kpa (6 to 7 psi) and a confining pressure of 6.9 to 13.8 kPa (1 to 2 psi). This is in accordance with other studies [11, 12], in which researchers recommended that the design *M*_*R*_ values for a confining pressure of 13.8 kPa (2 psi) and a deviatoric stress of 41.4 kPa (6 pi) should be considered. Therefore the stress levels in the base and subgrade may differ and should be considered separately in the laboratory in order to obtain reasonable results.

Two types of overall statistical analyses [13] were employed for the soil modulus: (1) ANOVA (analysis of variance) testing, which makes a comparison between the mean values and variances in different deviator stresses and (2) a method based on the *Z*-test, which specifies confidence intervals (CIs) that provide designers with more reliable design parameters as well as mean and standard deviation. A CI is a type of interval estimate of a population parameter and is used to indicate the reliability of an estimate. If CIs are constructed across many separate data analyses of repeated (and possibly different) experiments, the proportion of such intervals that contain the true value of the parameter will match the confidence level, which is the percentage of all possible samples that can be expected to include the true population parameter.

### 3.3. ANOVA (Analysis of Variance)

The ANOVA process is a method that allows for better understanding of the differences between two population means and the ratio of two population standard deviations. The statistical significance of a factor (*P* value) indicates whether there exists a significant mean difference between two analysis methods. First, before performing the test, the assumption is made that the data are normally distributed. Second, a hypothesis is developed based on the two methods being equal, and researchers test this hypothesis. For example, if the *P* value is greater than the critical alpha (i.e., 0.05), the probability of making the least favorable type of error, then the researchers have enough evidence to accept the given hypothesis.

### 3.4. *Z*-Test for Confidence Interval

Collected samples are usually limited; therefore, the true value of a sample is difficult to obtain. Researchers usually will not know the true value of a mean from sampling; rather, researchers would select a single random sample and construct the associated certain (i.e., 95%) CI in which the true value of the population parameters can be contained. Therefore, engineers can pick the safer parameter for the design purpose at cost effectiveness with confidence in the statistical procedure. *Z*-tests allow the endpoints of intervals to be computed based on sample information. Larger samples generally provide more information about the target population than do smaller samples. Therefore, the more samples that are collected, the greater the confidence in the findings and results obtained. Also, for a given sample size, the width of the CI for a parameter increases as the confidence coefficient increases. On the basis of this theory, the more soil data that is collected in the database, the more confidence engineers have in the evaluation of the soil modulus (or regression parameters).

### 3.5. Mechanical Properties of Subgrade for Design Level One

The MEPDG requires mechanical material properties as input to the constitutive relationships incorporated in these models to calculate material response and damage properties. For unbound base and soil materials, the resilient modulus (*M*_*R*_) is an important factor and is determined through cyclic load triaxial testing. In this advanced level, the MEPDG requires *k*_1_, *k*_2_, and *k*_3_ as inputs to characterize unbound material parameters. The measured *M*_*R*_ values at different confining and deviator stress are plotted, and the parameters are determined by regression analysis. The *M*_*R*_ is calculated by the following equation (3) and is being adapted in NCHRP 1-37A [2, 14]:

(3) $$\begin{array}{c} M_{R}=k_{1}p_{a}{\left(\frac{\theta }{p_{a}}\right)}^{k_{2}}{\left(\frac{\tau_{\text{oct}}}{p_{a}}+1\right)}^{k_{3}}, \end{array}$$

where *k*_1_, *k*_2_, and *k*_3_ = multiple regression constants evaluated from resilient modulus tests, *p*_*a*_ = atmospheric pressure = 14.7 psi (101.5 kPa), *θ* = bulk stress = *σ*_1_ + *σ*_2_ + *σ*_3_ = *σ*_*d*_ + 3*σ*_3_, *σ*_3_ = confining pressure, and *τ*_oct_ = octahedral shear.

Coefficient *k*_1_ is directly proportional to Young's modulus; it is a positive value. *k*_2_ should also be positive, since increasing the bulk stress produces a stiffening effect on the material. *k*_3_ is negative, since increase of shear produces a softening effect on the material, which results in lower *M*_*R*_ [15]. Therefore, soil samples that gave negative values for *k*_1_ and *k*_2_, or positive values for *k*_3_, were not used in the regression analysis. Equation (3) is applicable for all unbound materials, and it incorporates the effects of both deviatoric and volumetric stresses on *M*_*R*_, The standard laboratory methods for modulus testing are NCHRP 1-28A and AASHTO T307-99 [10]. For comparison, values of *k*_1_, *k*_2_, and *k*_3_ for different materials are summarized in Table 3. This table lists three typical soils at the optimum moisture content in Indiana, which are A-4, A-6, and A-7-6 on the basis of 140 soil samples. The ANOVA process is performed for comparison of two independent populations. It is a method that allows for better understanding of the differences between two population means and the ratio of two population standard deviations. The statistical significance of a factor (*P* value) indicates whether there exists a significant mean difference between the two analysis methods. First, before performing the test, the assumption is made that the data are normally distributed. Second, a hypothesis is developed based on the two methods being equal, and researchers try to test and reject this hypothesis. For example, if the *P* value is greater than the critical alpha (i.e., 0.05), the probability of making the least favorable type of error, then the researchers have enough evidence to accept the given hypothesis. ANOVA results (*P* value = 0.46) show that there is no significant difference at different deviator stresses (2 psi, 4 psi, and 6 psi) with a constant confining stress of 2 (or 4 psi). However, at the average, the modulus values show a 4% difference. On the other hand, ANOVA shows that the difference in resilient modulus values for confining stress was significant for all three soil types (A-4, A-6, and A-7-6 (*P* value = 0.01)). Therefore, accurate confining stress is important to decide the resilient modulus of cohesive soils. At the same time, it was found from test results that even when the materials were classified into the same type, variation of the parameters was quite large. This indicated that pavement evaluation at a certain site should be based on actual test results to reflect a local condition of pavement foundation materials.

Table 3 also lists the CI level for all three soils: with a 95% CI level, it was found in A-4 soil that the coefficient *k*_1_ layer coefficient (LC) values ranged from 289.25 to 391.59, with an average value of 333.44; the *k*_2_ values ranged from 0.37 to 0.6, with an average value of 0.45; and the values of *k*_3_ coefficients ranged from −0.38 to −0.18, with an average value of −0.28. In order to further examine suitability of the model parameters proposed in this study, measured *M*_*R*_ values obtained from the laboratory testing were compared with those using the proposed equation (1). The laboratory tests conducted on 126 subgrade soil samples to independently verify the prediction models show that the developed models predict *M*_*R*_ values close to the laboratory determined *M*_*R*_ values.

Due to limited space, Figure 3 lists only the measured and predicted resilient in confining level of 2 psi and deviator stress of 6 psi. Prediction models for the *k* coefficients in the generalized constitutive model for *M*_*R*_ were developed for AASHTO soil types A-4, A-6, and A-7-6 using multiple linear regression on data taken from the INDOT database. It can be found that they are evenly distributed around the line of equality with an *R* ^2^ value of 0.72. A plot of predicted and measured *M*_*R*_ values in Figure 3 also show that 31.46% and 51.74% of predicted *M*_*R*_ values fall within ±10% and 20%, respectively, of the laboratory *M*_*R*_ values. It can be concluded that the regression factors *k*_1_, *k*_2_, and *k*_3_ can provide relatively accurate inputs for level 1 of MEPDG. This is important to achieve since the MEPDG procedure includes terms for reliability and variability, which account for scatter in the data and use the estimated values to calculate pavement performance model. The reason could be (1) *k*_1_, *k*_2_, and *k*_3_ are universal regression coefficients for all confine and deviate stress levels and therefore these factors are only the best estimation in general seniors or (2) fine soils of A-4, A-6, and A-7-6 do not have clear trends corresponding to different stress, and because coefficients are hard to fit the laboratory testing results, it is found that, in individual laboratory test for a particular sample, the *R* ^2^ values associated with the *k*-coefficient regression equations range from 0.45 to 0.98.

#### 3.5.1. Unbound Material

The moisture sensitivity of an unbound coarse-grained material depends on the amount and nature of its fine fraction. Gravels and sands classified as GW, GP, SW, and SP are not likely to exhibit moisture sensitivity due to the absence of a sufficient number of the small pores necessary to create significant suction-induced effective stresses even at low moisture contents. The fine of number 53 stone, according to INDOT specifications, has only a 5%–10% moisture content. Therefore this study did not take into account moisture effects on the granular materials. Granular materials generally show highly nonlinear stress-strain behavior after the initial linear elastic range at small strains [16], and the testing conducted appeared to confirm a relationship between modulus, deviator stress, and confining pressure. When confining pressure increases, it yields both gravel and crushed stone modulus increase. In this study triaxial tests were conducted extensively on unbound material mixtures such as gravel and number 53 crush stone [17] widely used in Indiana. The materials were subjected to various levels of stresses depicting typical in situ conditions.  Figure 4 plots the resilient modulus at different confining and deviator stresses. The results show that the main effects of both stresses are significant. Figures 4 and 5 indicate that it is true that the higher the stress level, the higher the modulus value. Also, confining stresses show more influences on resilient modulus than deviator stresses do. Incorrect confining stress would lead to wrong base modulus. This finding is different from that of cohesive fine grain soil, in which deviator stresses have a small effect on resilient modulus compared to confining stresses. This may indicate that unbound materials have different mechanical properties, and AASHTO's suggestion that the granular base modulus is 207 kPa (30 psi) may be reasonable based on Figure 1 results under statics overburden and traffic loading.

One of the most widely utilized relationships for unbound granular base is the one proposed by Hicks and Monismith [18] as follows:

(4) $$\begin{array}{c} M_{R}=k_{1}\theta^{k_{2}}, \end{array}$$

where *M*_*R*_ is the resilient modulus in units of psi for the material subject to a bulk stress *θ*. The bulk stress *θ* is the sum of the principal stresses (*θ* = *σ*_1_ + *σ*_2_ + *σ*_3_). In repeated load triaxial compression tests, *θ* is the sum of the deviator stress and three times the confining stress (*θ* = *σ*_*d*_ + 3*σ*_3_). The constants *k*_1_ and *k*_2_ are material properties determined from data obtained in a laboratory test procedure, such as AASHTO T-307 [9].

Table 4 lists the regression coefficients for the nonlinear model and MEPDG model. It is found that both *R* ^2^ are 99%, indicating that the two models have very good fitness. Since *k*_1_ is related to material strength, it indicates that the crushed stone has better strength than gravel does. In addition, *k*_1_ with 5% fine is higher than that with 10% fine, which in general indicates that fines can affect the granular modulus in the base material. However, the values of *k*_2_ and *k*_3_ with 5% and 10% fines are very similar. This indicates that 5%–10% fines in the base materials affect the bulk stress (*k*_2_) and softening effect (*k*_3_) is not clear as the strength (*k*_1_). The same conclusion is made for crushed stone. As a result of the comparison, the crushed stone is recommended for use in the base material.

### 3.6. Mechanical Properties of Subgrade for Design Level Two

While it is expected that resilient modulus testing is to be completed for level 1 design, the cyclic load triaxial test on unbound/subgrade materials is complex, expensive, and time-consuming, and it requires well-trained personnel and expensive laboratory equipment. Therefore the resilient modulus test is not widely available. A level 2 design can be selected when laboratory *M*_*R*_ testing is not available. The value of resilient modulus can be obtained using typical correlations between resilient modulus and physical soil properties (i.e., dry unit weight, Atterberg limits, and specific gravity) or between resilient modulus and strength properties (i.e., CBR and confined compressive strength).

Level 2 design provides an intermediate level of accuracy. In this level 2 design, the MEPDG software allows users to input values of *M*_*R*_ that have correlations to local knowledge and experience and use EICM to adjust it for the effect of seasonal climate (i.e., the effect of freezing, thawing, etc.). Many states have been using FWD for backcalculating the subgrade soils. Thus, MEPDG level 2 inputs are expected to be used more commonly by INDOT for unbound and subgrade soil material characterization. This study evaluates the MEPDG current level 2 subgrade material characterizations based on the backcalculated modulus and using correlations with physical properties of tested soils.

### 3.7. Mechanical Properties of Subgrade for Design Level Three

For design level 3, only a typical representative *M*_*R*_ value at optimum moisture content is required. EICM is used to adjust the representative *M*_*R*_ for the seasonal effect of climate. Pavement designers may select the representative *M*_*R*_ value without the results being affected by EICM. This involves setting default values for the parameter based on the material class. These values also can be obtained based on soil classification or local experience. Such values are provided in the MEPDG from the mean of the soil database. The NCHRP study recommends that these default values be used in level 3 inputs.

### 3.8. FWD Test Site and Its Backcalculation

Falling weight deflectometers (FWDs) can be used to determine the moduli of pavement layers by an impulse load on the surface and to measure deflections with geophones. Tests were conducted in the driving lanes in both directions at 100-meter intervals. Based on previous INDOT studies and experiences, a minimum of 16 testing locations per mile is adequate to provide statistically sound analysis. Three drop load levels consisting of 7 kip, 9 kip, and 11 kip were used. Only the 9-kip load level was used for the analysis. For each test, the pavement surface deflections were measured at the distance of 0, 8.0, 12.0, 18.0, 24.0, 36.0, 48.0, and 60.0 inches from the center of the load area. 1993 AASHTO recommends using the following formula for determining the resilient modulus value of the subgrade soil based on the deflection measurements (1):

(5) $$\begin{array}{c} M_{R}=\frac{0.24P}{d_{r}r}, \end{array}$$

where *M*_*R*_ = subgrade resilient modulus (psi), *P* = applied load (pounds), *d*_*r*_ = deflection at a distance *r* from the center of the load (inches), and *r* = distance from center of load (inches).

## 4. Results and Discussion

### 4.1. Comparison between Lab and Backcalculated Resilient Modulus

The testing program consisted of both field and laboratory tests. Four roads with existing asphalt pavements across Indiana were chosen for this study. Test sites were chosen to represent typical subgrade material throughout Indiana. A map of these sites is shown in Figure 6. Four roads including US 27, SR 32, SR 69, and test road in the INDOT research office were selected. Each road has three testing sites and each site has 100-meter. Subgrades at these sites mostly consisted of A-4 and A-6 soils. As mentioned previously, the objective of this study was to construct relationships between the laboratory *M*_*R*_ and monthly or seasonal in situ *M*_*R*_ obtained from the FWD test for typical subgrade materials. For example, laboratory *M*_*R*_ (at OMC) = FWD *M*_*R*_ × factor, in which factor is the function of moisture content, temperature, and so forth. Disturbed soil samples were collected at two locations from each section. The following laboratory tests were performed to evaluate soil index properties: (a) specific gravity (*G*_*s*_) and water content (*w*%) tests; Atterberg limit tests; (b) hydrometer tests for grain size distribution; and (c) compaction tests.

The AASHTO Design Guide (1986, 1993) [1] suggests that the backcalculated moduli are approximately 3 times higher than the resilient modulus obtained from the triaxial load resilient modulus test. Disturbed soil samples were collected at two locations from each section. The following laboratory tests were performed to evaluate soil index properties: (a) specific gravity (*G*_*s*_) and water content (*w*%) tests; (b) Atterberg limit tests; (c) hydrometer tests for grain size distribution; and (d) compaction tests. Results of these tests are shown in Table 5.

A previous study [19] showed that if the roadbed soil samples were tested in the laboratory at similar water contents as the field water contents at the time when the FWD tests were conducted, then the ratios of the backcalculated to the laboratory-obtained modulus values are close to 1. However, our finding is similar to those reported in the literature, where the ratio between the backcalculated and the laboratory-determined *M*_*R*_ values vary from almost 1.6 to almost 5.0:

(6) $$\begin{array}{c} \text{Lab}\;\;M_{R}\left(\text{at}\;\;\text{OMC}\right)=\text{FWD}\frac{M_{R}}{4}. \end{array}$$

The results obtained show that the average FWD backcalculated moduli are approximately 4 times higher than the laboratory resilient moduli. This result is close to the recommendations of AASHTO, but the large scatter in these values suggests that there is no clear relationship between the two. There are several possible reasons for this result. First, the FWD tests were performed on in situ conditions whereas the resilient modulus tests were performed on soil samples at OMC conditions and certain stress boundary conditions. Second, the FWD tests were performed at different times of the year, causing variations in moisture content of the soil, which affects the FWD modulus. Third, the stress calculations for the FWD test were based on a multilayer-elastic analysis, while the pavements are not elastic. For each soil classification, Table 6 provides a list of the average backcalculated *M*_*R*_ value of the subgrade beneath flexible pavement, and the ratios between the two sets of averages are also listed in Table 5.

### 4.2. Moisture and Seasonal Effects

During the construction stage, pavement materials are typically compacted to over 95% of optimum densities. However, the moisture and densities of the pavement structure will change with time, due to environmental and traffic factors. The in situ moisture content and densities of the soils were collected from the field test program. Using the same soils obtained from the field, the modified proctor compaction tests were conducted in the laboratory to determine the OMC and maximum dry densities.

The moisture content of most cohesive soil materials has been found to affect the resilient response characteristics of the material in both laboratory and in situ conditions. A previous study [20] shows that the behaviors of these materials at high degrees of saturation have all shown a notable dependence of resilient modulus on moisture content. With the modulus decreasing with growing saturation level it showed a significant reduction of resilient modulus of soils as the moisture content was increased above the optimum moisture content. The triaxial tests following the AASHTO T307-99 [10] procedure were conducted on the A-4, A-6, and A-7-6 cohesive soils compacted at optimum water content and at 2% above the optimum. The researchers did not perform the cyclic load triaxial testing (CTT) at 2% below the optimum because testing of OMC is critical and it shows how resilient modulus drops with an increase in moisture. Secondly, some tests stopped because samples are too dry. The measured resilient modulus for A-4 and A-6, A-7-6 soils, along with their respective standard deviations and coefficients of determination *R* ^2^, is presented in Table 7 and Figure 7. It is observed that with an increase of 2% in OMC, the resilient modulus decreases as much as 4 times. A coefficient of *k*_1_ value, a factor that is proportional to resilient modulus, changed dramatically compared to *k*_1_ in Table 3. *k*_2_ and *k*_3_ also changed compared to those values in Table 3. The value of *k*_1_, proportional to Young's modulus, decreased as much as 40% between OMC and 2% + OMC. The contents of fine in A-4, A-6, and A-7-6 are 15.79%, 22.29%, and 32.76%, respectively. The main reason is that the soil contains certain amounts of fines, and it indicates that an increase in moisture content causes significant degradation of the resilient modulus of cohesive soils.

Seasonal adjustment factors for the subgrade soil were estimated for each site at Indiana. Seasonal timing for the selected four seasons (summer, fall, winter, and spring) were also determined for the different sites based on the average monthly rainfall and air temperature. FWD *M*_*R*_ at all test sites increases when early summer and winter months are compared. In terms of the time of the year, resilient modulus of subgrade is typically 1.2 to 4 times higher in the coldest months (December, January, and February) as compared to the rest of the year [21]. The results obtained from this study show that

(7) Average  Dec.  FWD  MR  =1.64  Average  May  FWD  MR  (US  27)Average  Dec.  FWD  MR  =1.16  Average  May  FWD  MR  (SR  32)Average  Dec.  FWD  MR  =1.57  Average  May  FWD  MR  (SR  69)Average  Dec.  FWD  MR  =1.20  Average  May  FWD  MR  (test  road).

Resilient modulus also becomes substantially lower in the thawing period of March and April. The melted ice fully saturates the soil and the soil reaches its weakest state [22]. Resilient modulus changes with variation in the moisture content. It is highest at OMC and decreases at higher or lower moisture contents. In April and May, due to the melting of ice, the moisture content of the subgrade increases and saturates the soil. This leads to a lower FWD *M*_*R*_ value. As the moisture begins to drain out in the months ahead, the subgrade moduli increase again and reach their peak in the months of December and January. Varying precipitation can also affect the subgrade moisture content, thus affecting the resilient moduli, but the effect of precipitation on moisture content of subgrade is not substantial [19]. This trend is properly shown in Figure 8, which illustrates the gradual increase in the FWD *M*_*R*_ from April to December. Results show that on average the FWD *M*_*R*_ increases by approximately 40% from May to December.

### 4.3. Relationship between Coefficients and Material Properties

The correlation equations described herein were developed using regression analyses. Since the form of *M*_*R*_ = *f* (*σ*_*d*_, *σ*_3_, other *σ* expressions, *k*_1_, *k*_2_, *k*_3_,…, *k*_*i*_) in which the *k*_1_, *k*_2_, and *k*_3_ parameters are correlated to soil properties. The correlations are created by conducting a series of resilient modulus tests on various soils and analyzing the results of each test with parameter models. The *k*_1_, *k*_2_, and *k*_3_ parameters are then determined for each test and are referred to as “measured” parameters. By correlating the measured parameters to soil properties (e.g., LL, PI, % CLAY, % GRAV, % SILT, etc.), the resilient modulus of other similar soils can be estimated at a variety of stress states without conducting another laboratory test.

One hundred twenty-six soil samples were collected to obtain the *k* coefficient for AASHTO category soil (A-4, A-6, and A-7-6) with known laboratory *M*_*R*_ value using (3). A previous study [3, 4] shows that material constants or regression coefficients can be estimated from soil index properties. Kim and Siddiki [7] reported a reasonably strong correlation with an *R* ^2^ value of 0.847 while predicting material constants for the octahedral model using twelve soil parameters. Results conducted by Mohammad et al. [23] showed that specific soil types have good statistical relationships. After obtaining *k*_1_, *k*_2_, and *k*_3_ for each soil sample collected for a soil type, prediction models for the *k* coefficients were developed using the multiple linear regression technique and were carried out to relate these individual soil sample *k* coefficient values with the overall physical properties of a particular soil type and obtain a single set of *k*_1_, *k*_2_, and *k*_3_ prediction equations applicable to that particular soil type. The *R* ^2^ value in the regression modeling was highly correlated with the soil properties; it is as high as 0.99, and as low as 0.79. This indicates that the proposed method is a very efficient way to predict the MEPDG inputs.

The soil properties that were considered for this study included the following: ADDO (actual dry density at OMC (pcf)) and AMCO (actual moisture content at OMC%), % CLAY (percent clay in particle size distribution curve), % GRAV (percent gravel in particle size distribution curve), LL (liquid limit), MDD (max. dry density), OMC (optimum moisture content), PI (plasticity index), % SAND (percent sand in particle size distribution curve), % SILT (percent silt in particle size distribution curve), and SG (specific gravity). A nonlinear regression, a list of models, was performed using the RSQUARE selection method available in the Statistix 8 program [24]. The regression coefficients in the *M*_*R*_ predictive model are summarized in Table 8, along with their respective coefficients of determination *R* ^2^. For example, *k*_1_ for A4 can be expressed as *k*_1_ = 15.2755 × ADDO + 102.276 × AMCO + 15.5439 × % CLAY + 11.5423 × % GRAV − 2.68004 × LL − 30.39 × MDD − 127.734 × % OMC − 14.5558 × PI + 12.5928 × % SAND + 10.2289 × % SILT + 562.592 × SG.

In order to verify the prediction models developed herein, some samples of A-4, A-6, and A-7-6 soil types were tested in the laboratory to determine *M*_*R*_ using AASHTO standards. The parameters are listed in Table 8. The laboratory tests have been mentioned and included repeated load resilient modulus tests, determination of moisture content and density of the soil specimen used for the *M*_*R*_ test, sieve analysis, Atterberg limits tests, and proctor tests. All soil samples were compacted at OMC for *M*_*R*_ testing as obtained from proctor tests. To determine the predicted values of *M*_*R*_, values of the soil properties obtained from the laboratory tests were substituted in the corresponding prediction equations of *k* coefficients for each of the soil types presented in previous sections. Then, these *k*-coefficient values were substituted into the equation listed in Table 8. The laboratory and predicted *M*_*R*_ values for the A-4, A-6, and A-7-6 soil samples are compared. An analysis of the *M*_*R*_ values showed that 93.52%, 90.83%, and 94.33% of *M*_*R*_ values obtained from the prediction equations for A-4, A-6, and A-7-6, respectively, fell within ±10% of the measured *M*_*R*_ values for the corresponding soil type.

## 5. Conclusions

On the basis of the study presented in this paper the following conclusions can be drawn.

1. Resilient modulus is an excellent measurement under pavement materials service condition in the pavement structure. If the test is properly performed, the resilient modulus measurement is reliable for inputs of the MEPDG. Material properties can be used to predict the resilient modulus, its *R* ^2^ values ranging from 0.79 to 0.97.
2. Backcalculated modulus from FWD data provides a practical alternative for inputs of level 2 designs. Backcalculation from in situ test device measurements and estimation using correlations with physical properties of tested soils can be employed to predict resilient modulus. Correlation equations have been developed with more commonly to estimate the resilient modulus of the unbound materials and cohesive soil.
3. The mechanistic analysis performed using elastic layer theory shows that the resilient modulus under a state of stress with a confining pressure of 13.8 kPa and 27.6 kPa is representative for the resilient behavior of base and subgrade soil material in flexible pavements, respectively. The confining stresses statistically influence resilient modulus for granular and cohesive subgrade soils.
4. Backcalculated moduli herein are similar to the NCHRP recommended in situ resilient modulus. On the other hand, on average, the in situ modulus from FWD testing is about 4 times higher than the laboratory resilient modulus of the soil compacted at OMC. Therefore adjusted factors are needed if laboratory testing is input in the MEPDG.
5. The variation of the subgrade modulus and moisture followed the rule that the modulus decreased with moisture increase. This conclusion was valid for all soils in which the laboratory moisture contents were above the optimum. On the other hand, it is believed that the increase in modulus with increase in moisture would be reasonable if the existing moisture condition is on the dry side. Thus, an increase in moisture will result in a higher modulus until it reaches the optimum, and then it starts to decrease.
6. Seasonal factors cannot be ignored because winter FWD modulus is on average approximately 40% higher than early summer FWD modulus. The in situ back-calculated modulus at most of the Indiana sites showed that it has only a small seasonal fluctuation compared to the moisture effect on modulus in the laboratory testing. It may prove that an in situ finding is quite different from the laboratory finding. The observed seasonal variation could be related to the rainfall amount, the ground water level (GWL), or the soil type (fine or coarse, plastic or non-plastic). The further investigation will be needed.
7. Prediction models for the *k* coefficients in the generalized constitutive model for *M*_*R*_ were developed for AASHTO soil types A-4, A-6, and A-7-6 using multiple linear regressions on data taken from the INDOT database. The *R* ^2^ values associated with the *k*-coefficient regression equations range from 0.92 to 0.93 for A-4, from 0.79 to 0.99 for A-6, and from 0.90 to 0.99 for A-7-6 soil.

## Figures and Tables

**Figure 1:** Stress level at the middle of the base.

**Figure 2:** Stress level at the top of the subgrade.

**Figure 3:** Measured versus predicted resilient modulus values at different confining and deviator stresses (*R* ^2^ = 0.72).

**Figure 4:** Laboratory resilient modulus for unbound materials at different confining and deviator stresses.

**Figure 5:** Laboratory resilient modulus for gravel and crush stone at bulk stress.

**Figure 6:** Existing pavements.

**Figure 7:** Modulus variation and moisture content of soil (*σ*_*c*_ = 2 psi and *σ*_*d*_ = 6 psi).

**Figure 8:** Seasonal variation of FWD *M*_*R*_ in test road.

**Table 1:** Basic statistical parameters for soil samples.

Soil samples	Soil type		LL	PI	Specific gravity	Max. dry density pcf	OMC %	Actual Dry Density at OMC pcf	Actual moisture content at OMC pcf
29	A-4	Min.	15.5	6.2	2.66	109	13.8	107.9	15.2
		Max.	34.6	10	2.75	129.9	19.3	130.4	19.1
		Mean	26.5	7.2	2.66	115.1	14.2	112.7	14.3
		Standard deviation	5.3	2	0.05	9	3.4	9.9	3.4

69	A-6	Min.	23	5.8	2.54	104.1	10.8	102	10.6
		Max.	40	26	2.76	125.7	19.5	124.7	19.8
		Mean	33.1	15.3	2.67	113.3	15.3	111.6	15.4
		Standard deviation	4.3	3.6	0.04	5.4	2.2	5.2	2.2

28	A-7-6	Min.	41	16.7	2.62	92.2	14.4	89.9	14.4
		Max.	78	55	2.77	114.5	29	113.6	29.1
		Mean	46.9	26	2.7	105.6	19.1	103.9	19.3
		Standard deviation	8.3	8	0.04	5.9	3.4	6.3	3.3

**Table 2:** Range of pavement cross section and material properties used in sensitive analysis.

AC courses/layers	Thickness (m)	Modulus (kpa)	Poisson's ratio	Density (kg/m^3^)
HMA	0.1, 0.13, 0.15, 0.18, 0.2	3450	0.35	2400
Combination of base and subbase	0.2, 0.23, 0.26, 0.28, 0.3	207	0.40	2080
Roadbed soil	Infinite	34.5, 69	0.45	1920

**Table 3:** MEPDG Level 1 for different cohesive soils (*σ*_*c*_ = 2 psi, *σ*_*d*_ = 6 psi).

Soil type		*k*_1_ at OMC	*k*_2_ at OMC	*k*_3_ at OMC
A-4	Lower level	289.25	0.37	−0.38
	Upper level	391.59	0.6	−0.18
	Mean	333.44	0.45	−0.28
	Standard deviation	102.9	0.25	0.19

A-6	Lower level	270.68	0.28	−0.31
	Upper level	317.62	0.37	−0.22
	Mean	294.15	0.33	−0.26
	Standard deviation	67.27	0.13	0.13

A-7-6	Lower Level	297.42	0.13	−0.28
	Upper level	361.89	0.27	−0.15
	Mean	329.66	0.21	−0.22
	Standard deviation	60.5	0.12	0.12

Note: 1 psi = 6.9 kPa.

**Table 4:** *k*-*θ* Model versus MEPDG Model.

		*k*-*θ* Model				MEPDG Model				
		*k*_1_	*k*_2_	*R* ^2^	Adj *R* ^2^	*k*_1_	*k*_2_	*k*_3_	*R* ^2^	Adj *R* ^2^
Gravel	5% fine	2852.44	0.58176	0.9758	0.974	698.135	0.72883	−0.15741	0.9934	0.9923
	10% fine	2664.44	0.5778	0.9772	0.9754	643.1336	0.72655	−0.15921	0.9954	0.9946

Crushed stone	5% fine	2426.56	0.62827	0.9737	0.9717	635.3096	0.80524	−0.18942	0.9955	0.9947
	10% fine	1334.471	0.76537	0.9662	0.9636	506.1193	0.94124	−0.18825	0.9805	0.9773

**Table 5:** Material properties for soils used.

Site	Sample	AASHTO	USCS	F200	Liquid limit	Plastic limit	Plasticity index	Specific gravity	Optimum moisture content	Maximum dry density (pcf)
US 27	85.00	A-6	CL	77.1%	34.8%	20.8%	14.1%	2.55	14.8%	115.4
	85.06	A-6	CL	65.7%	27.2%	17.0%	10.2%	2.58	15.5%	117.3
	85.36	A-4	CL-ML	72.3%	22.6%	15.8%	6.9%	2.57	12.9%	118.6
	85.42	A-4	CL	64.0%	23.6%	15.9%	7.7%	2.71	13.0%	118.6
	85.78	A-4	CL-ML	72.9%	28.9%	22.1%	6.8%	2.55	16.8%	110.4
	85.84	A-4	ML	78.4%	36.4%	27.1%	9.3%	2.64	19.6%	107.0

SR 32	58.60	A-4	ML	55.2%	37.4%	26.8%	10.6%	2.96	17.5%	108.0
	58.66	A-4	ML	57.4%	27.5%	24.3%	3.2%	3.14	15.3%	109.8
	59.14	A-4	CL	57.5%	33.2%	24.1%	9.0%	2.75	15.0%	118.6
	59.20	A-6	CL	80.3%	40.3%	23.3%	17.0%	2.70	19.0%	108.6
	59.68	A-4	SC	47.5%	30.5%	21.2%	9.3%	2.75	13.2%	120.4
	59.74	A-4	ML	56.2%	29.1%	25.3%	3.8%	3.05	15.5%	122.3

SR 69	27.00	A-4	ML	90.9%	25.5%	24.8%	0.7%	2.81	17.3%	104.8
	27.06	A-4	CL	94.2%	30.7%	21.6%	9.1%	2.48	16.2%	111.7
	28.01	A-4	CL	52.3%	26.7%	19.4%	7.3%	2.67	14.9%	115.4
	28.07	A-4	ML	83.5%	25.1%	23.1%	1.9%	2.82	15.5%	111.7
	29.04	A-1-b	SM	24.2%	19.4%	18.5%	0.9%	2.73	7.5%	124.8
	29.10	A-4	ML	60.7%	19.4%	16.4%	3.0%	2.66	10.3%	123.6

Test Road		A-4	CL	63.7%	30.6%	21.4%	9.1%	2.68	15.4%	109.6

**Table 6:** Comparison between lab and backcalculated resilient modulus.

AASHTO classification	OMC (%)	Lab *M*_*R*_ (kpa)	Backcalculation *M*_*R*_ (kpa)	Reduction factor
A-4	14.25	61893	247779	4.00
A-6	15.42	39564.6	128133	3.24

**Table 7:** MEPDG Level 1 for 2% + OMC.

Soil Type		*k*_1_ at 2% + OMC	*k*_2_ at 2% + OMC	*k*_3_ at 2% + OMC
A-4	Lower level	184.99	0.23	−0.37
	Upper level	246.63	0.44	−0.10
	Mean	219.31	0.32	−0.19
	Standard deviation	72.18	0.24	0.27

A-6	Lower level	159.17	0.25	−0.35
	Upper level	183.00	0.34	−0.25
	Mean	169.8	0.28	−0.30
	Standard deviation	45.49	0.18	0.17

A-7-6	Lower level	169.89	0.12	−0.43
	Upper level	258.42	0.32	−0.26
	Mean	219.25	0.21	−0.34
	Standard deviation	91.7	0.21	0.17

**Table 8:** Correlation between MEPDG inputs and soil properties at OMC.

Soil type	A4			A-6			A-7-6		
MEPDG inputs	*k*_1_	*k*_2_	*k*_3_	*k*_1_	*k*_2_	*k*_3_	*k*_1_	*k*_2_	*k*_3_
ADDO	15.2755	−0.0537	0.05003	−10.373	−0.01986	−0.01523	40.4804	−0.09401	0.13677
AMCO	102.276	0.38034	0.53396	−160.526	0.01833	−0.00001	−71.9733	0.41507	−0.16641
CLAY	15.5439	−0.00158	−0.00486	−1.23003	−0.00484	0.00908	13.5356	0.06418	−0.03009
GRAVEL	11.5423	−0.00577	−0.01169	−1.41065	−0.01011	0.01576	14.7768	0.0352	−0.02735
LL	−2.68004	0.05675	0.04337	14.3789	−0.00358	−0.00555	3.28479	−0.02432	0.00768
MDD	−30.39	0.07329	−0.11358	0.66964	0.02925	0.00598	−46.8996	0.0268	−0.11805
OMC	−127.734	−0.41051	−0.68651	123.671	−0.01324	−0.02212	43.007	−0.50741	0.18766
PI	−14.5558	0.03855	0.025	6.63765	−0.00985	0.01139	5.8166	0.02229	−0.00922
SAND	12.5928	0.01153	−0.00194	4.59136	−0.00646	0.0116	15.0582	0.09066	−0.03127
SILT	10.2289	0.00322	−0.00836	2.00541	−0.00263	0.00892	19.0182	0.07255	−0.02671
SG	562.592	−1.38553	3.25546	469.806	−0.06798	0.06054	−115.307	0.81695	0.15138
*R* ^2^	0.97	0.92	0.93	0.95	0.88	0.79	0.99	0.90	0.95

Note: CLAY = particles smaller than 0.002 mm.

GRAVEL = particles from 3 in (75 mm) to NO 10 (2 mm) sieve.

SAND = particles from passing NO 10 (2 mm) to NO 200 (75 *μ*m) sieve.

SILT= particles from 0.075 to 0.002 mm.
